# Radiotherapy after surgery has significant survival benefits for patients with triple‐negative breast cancer

**DOI:** 10.1002/cam4.1954

**Published:** 2019-01-10

**Authors:** Yi Yao, Yuxin Chu, Bin Xu, Qinyong Hu, Qibin Song

**Affiliations:** ^1^ Cancer Center Renmin Hospital of Wuhan University Wuhan China

**Keywords:** radiotherapy, surgery, survival, triple‐negative breast cancer

## Abstract

**Objectives:**

The value of adjuvant radiotherapy for triple‐negative breast cancer (TNBC) has been controversial recently. This study aims to clarify the influence of radiotherapy on the survival of TNBC patients after surgery based on a large population analysis.

**Methods:**

The Surveillance, Epidemiology, and End Results (SEER) database was exploited to select eligible patients from 2010 to 2014. The categorical variables were examined by chi‐square tests. Breast cancer‐specific survival (BCSS) and overall survival (OS) were compared among patients who received or not received adjuvant radiotherapy after surgery by Kaplan‐Meier method with log‐rank test. Univariate and multivariate survival analysis of BCSS and OS were performed using the Cox proportional hazard model.

**Results:**

Totally 22 802 patients were enrolled in this study, of which 10 905 patients received radiotherapy after surgery while 11 897 patients did not receive radiotherapy. Compared with those patients who did not receive radiotherapy, the radiation group had a larger proportion of tumor size <2.0 cm (45.8% vs 38.8%) and chemotherapy (82.5% vs 67.4%). The Kaplan‐Meier plots displayed that patients in the radiation group had better survival than the no radiation group in both BCSS and OS (*P* < 0.001, respectively). In univariate Cox analysis of BCSS, age 40‐60, married status, white and other race, chemotherapy, radiation, and surgery were associated with better survival (HR < 1, *P* < 0.05). Specifically, patients who received radiotherapy exhibited better BCSS (HR = 0.52, 95% CI = 0.48‐0.57, *P* < 0.001). After adjusting for confounding factors by multivariable Cox regression analysis, receipt of radiotherapy was still associated with improved BCSS (HR = 0.79, 95% CI = 0.72‐0.87, *P* < 0.001). Survival analysis of OS produced similar results. Generally, these data indicate that radiotherapy after surgery has significant survival benefits for the TNBC patients.

**Conclusions:**

This study has confirmed the survival advantage of adjuvant radiotherapy for the TNBC patients. These findings may optimize the current individualized treatment decisions for this patient population.

## 1 INTRODUCTION

Triple‐negative breast cancer (TNBC) is a heterogeneous disease which represents 15%‐20% of breast cancer incidences.^1^ The incidence increased from 14.5 new cases per 10^5^ inhabitants in 1993 to 70.2 per 10^5^ in 2012.^2^ Compared with other subtypes, TNBC is associated with an early age at presentation, larger tumor sizes, higher rates of recurrence, more aggressive biology, and poorer prognosis.^3^ Particularly, the median survival of TNBC patients with brain metastasis was only 6 months.^4^ The absence of hormonal or targeted therapy against TNBC makes it a clinical challenge for oncologists in terms of patient management.^5^

Radiotherapy such as radiosurgery or hippocampal sparing technique may provide efficacious local tumor control with minimal side effects.^6^ However, controversies still exist with respect to the use of radiotherapy for patients with TNBC. The value of adjuvant radiotherapy on survival of TNBC patients after surgery is still uncertain. A recent study reported that women with T1‐2N0 TNBC treated with modified radical mastectomy without radiotherapy had a significantly increased risk of locoregional recurrence and poorer survival.^7^ On the other hand, another study revealed that omission of radiotherapy in patients with pN0 TNBC did not seem to result in poorer outcome.^8^ Those previous reports investigating the survival outcomes of TNBC patients according to local radiotherapy status have produced conflicting results. Some studies were underpowered because of their small sample sizes. Thus, accurately evaluating the role of radiotherapy in the prognosis of TNBC has become increasingly important.

The present study used the Surveillance, Epidemiology, and End Results (SEER) database to enroll a large population of TNBC cases to investigate the survival differences between radiation and no radiation groups, which may overcome the defects of previous studies. We have examined patient characteristics (age, marital status, and race), tumor variables (grade, TNM stage, and tumor size), and treatment (chemotherapy, radiation, and surgery). Breast cancer‐specific survival (BCSS) and overall survival (OS) were comprehensively compared between patients who received radiotherapy after surgery and those who did not receive radiation. We sought to evaluate factors associated with the prognosis of TNBC patients, highlighting the influence of radiotherapy on the survival outcomes of TNBC patients.

## 2 PATIENTS AND METHODS

### 2.1 Patient selection

All the data in this study were extracted from Surveillance, Epidemiology, and End Results (SEER) 18 registries Custom Data (with additional treatment fields). We used SEER*Stat version 8.3.5 software to retrieve data files directly. Given this database is publicly available and does not require informed patient consent, our study was exempted from ethical institutional review board. The inclusion criteria for the patients: (a) female unilateral breast cancer diagnosed from 2010 to 2014; (b) primary breast cancer as the first or only cancer diagnosis; (c) the breast cancer subtype was triple negative; (d) radiation sequence with surgery was “No radiation and/or cancer‐directed surgery” and “Radiation after surgery.” The diagnosis was not obtained from a death certificate or autopsy. Those patients with unknown marital status, race, grade, AJCC TNM stage were excluded. Patients before 2010 were excluded because HER2 status was not recorded in SEER until 2010. Those patients after 2014 were also excluded because the database only updated to 31 December 2014. The process of patient selection can be seen in Figure 1.

**Figure 1:** The flowchart of patients’ selection from the SEER database

### 2.2 Data collection

The following variables were collected from each patient: age at diagnosis, marital status, race recode, tumor grade, AJCC TNM Stage, tumor size, chemotherapy recode, radiation status, surgery type, SEER cause‐specific death classification, vital status, and survival months. BCSS was defined as the date from diagnosis to death from breast cancer. OS was defined as the period from diagnosis to death from any cause. BCSS was the primary endpoint, while OS was the secondary endpoint.

### 2.3 Statistical analysis

Demographic statistics included age at diagnosis, marital status, race recode. Age was divided into <40, 40‐60, >60 years groups. Marital status comprised married and not married including divorced, widowed, single (never married) and separated. Race recodes included white, black, and other (American Indian/AK Native, Asian/Pacific Islander). Tumor features included grade, AJCC TNM Stage, and tumor size. The therapy contained chemotherapy, radiation, and surgery. Chi‐square tests were used to evaluate the differences of categorical variables between no radiation and radiation groups. Associations between clinicopathological factors with receipt of radiotherapy after surgery were evaluated using logistic regression analysis. Kaplan‐Meier plots and log‐rank tests were adopted to compare the differences of BCSS and OS between the two groups. Univariate and multivariate Cox proportional hazard models were used to characterize factors for patients' survival, with hazard ratios (HRs) and 95% confidence intervals (CIs) indicated. All the statistical analyses were performed using SPSS statistical software, version 23.0 (SPSS, Chicago, IL, USA). A two‐tailed *P* < 0.05 was considered statistically significant.

## 3 RESULTS

### 3.1 Patient characteristics

According to the inclusion and exclusion criteria depicted above, totally 22 802 patients were enrolled in this study, of which 10 905 patients received radiotherapy after surgery while 11 897 patients did not receive radiotherapy. The demographics, tumor, and therapy characteristics in each group can be seen in Table 1. Except for grade, there were significant differences in many variables between the two groups. Compared with those patients who did not receive radiotherapy, patients in the radiation group were more 40‐60 years old (46.5% vs 43.7%), more married (59.1% vs 54.2%), more black race (21.8% vs 19.1%), more stage T1 (45.9% vs 38.7%) while less stage T2 (39.9% vs 44.5%), more N1‐N3 while less N0 (62.1% vs 65.6%), all the *P* < 0.001. Furthermore, the radiation group had a larger proportion of tumor size <2.0 cm (45.8% vs 38.8%) and chemotherapy (82.5% vs 67.4%). As for surgery type, 34.7% of the patients in the no radiation group received total mastectomy, while 71.5% in the radiation group received partial mastectomy (*P* < 0.001). The detailed patient characteristics are summarized in Table 1.

**Table 1:** Baseline characteristics of TNBC patients included in this study (n = 22 802)

Characteristics	Total, n (%) n = 22 802	No radiation, n (%) n = 11 897	Radiation, n (%) n = 10 905	*P*‐value
Age (y)				
<40	2479 (10.9)	1377 (11.6)	1102 (10.1)	<0.001
40‐60	10 267 (45.0)	5200 (43.7)	5067 (46.5)	
>60	10 056 (44.1)	5320 (44.7)	4736 (43.4)	
Marital status				
Not married	9909 (43.5)	5449 (45.8)	4460 (40.9)	<0.001
Married	12 893 (56.5)	6448 (54.2)	6445 (59.1)	
Race				
Black	4652 (20.4)	2275 (19.1)	2377 (21.8)	<0.001
White	16 422 (72.0)	8653 (72.7)	7769 (71.2)	
Others	1728 (7.6)	969 (8.1)	759 (7.0)	
Grade				
I	470 (2.1)	238 (2.0)	232 (2.1)	0.292
II	3876 (17.0)	2035 (17.1)	1841 (16.9)	
III	18 250 (80.0)	9504 (79.9)	8746 (80.2)	
IV	206 (0.9)	120 (1.0)	86 (0.8)	
Stage T				
I	9613 (42.2)	4610 (38.7)	5003 (45.9)	<0.001
II	9639 (42.3)	5291 (44.5)	4348 (39.9)	
III	2036 (8.9)	1064 (8.9)	972 (8.9)	
IV	1514 (6.6)	932 (7.8)	582 (5.3)	
Stage N				
0	14 573 (63.9)	7800 (65.6)	6773 (62.1)	<0.001
1	5665 (24.8)	2906 (24.4)	2759 (25.3)	
2	1431 (6.3)	624 (5.2)	807 (7.4)	
3	1133 (5.0)	567 (4.8)	566 (5.2)	
Stage M				
0	21 643 (94.9)	10 985 (92.3)	10 658 (97.7)	<0.001
1	1159 (5.1)	912 (7.7)	247 (2.3)	
Tumor size (cm)				
<2.0	9612 (42.2)	4618 (38.8)	4994 (45.8)	<0.001
2.0‐5.0	9631 (42.2)	5285 (44.4)	4346 (39.9)	
>5.0	3559 (15.6)	1994 (16.8)	1565 (14.4)	
Chemotherapy				
No/unknown	5787 (25.4)	3874 (32.6)	1913 (17.5)	<0.001
Yes	17 015 (74.6)	8023 (67.4)	8992 (82.5)	
Surgery type				
No surgery	1682 (7.4)	1613 (13.6)	69 (0.6)	<0.001
Partial mastectomy	11 165 (49.0)	3369 (28.3)	7796 (71.5)	
Total mastectomy	5095 (22.3)	4132 (34.7)	963 (8.8)	
MRM	4860 (21.3)	2783 (23.4)	2077 (19.0)	

Not married: Including divorced, widowed, single (never married), separated.

Others: Including American Indian/AK Native, Asian/Pacific Islander.

MRM, Modified radical mastectomy; TNBC, triple‐negative breast cancer.

### 3.2 Factors associated with receipt of radiotherapy after surgery

To better understand the criteria of patient selection, we further analyzed the clinicopathological factors associated with receipt of radiotherapy. As is vividly revealed in Table 2, the univariate logistic analysis demonstrated that age >40, married, stage N1‐N3, chemotherapy, and surgery were associated with increased propensity of receiving radiotherapy, compared to each referent group (OR > 1, *P* < 0.05). The multivariate logistic analysis indicated that patients who were married, stage T3‐T4, stage N1‐N3, received chemotherapy, and surgery were more liable to be treated with radiotherapy (OR > 1, *P* < 0.05).

**Table 2:** Factors associated with receipt of radiotherapy after surgery (n = 22 802)

Variables	Univariate logistic model		Multivariate logistic model	
	OR (95% CI)	*P* value	OR (95% CI)	*P* value
Age (y)				
<40	Reference		Reference	
40‐60	1.22 (1.12‐1.33)	<0.001	0.96 (0.86‐1.06)	0.425
>60	1.11 (1.02‐1.22)	0.018	1.03 (0.93‐1.15)	0.554
Marital status				
Not married	Reference		Reference	
Married	1.22 (1.16‐1.29)	<0.001	1.14 (1.07‐1.21)	<0.001
Race				
Black	Reference		Reference	
White	0.86 (0.81‐0.92)	<0.001	0.90 (0.83‐0.97)	0.007
Others	0.75 (0.67‐0.84)	<0.001	0.85 (0.74‐0.97)	0.015
Grade				
I	Reference		Reference	
II	0.93 (0.77‐1.12)	0.445	0.75 (0.60‐0.94)	0.011
III	0.94 (0.79‐1.13)	0.538	0.63 (0.51‐0.79)	<0.001
IV	0.74 (0.53‐1.02)	0.068	0.61 (0.41‐0.90)	0.013
Stage T				
I	Reference		Reference	
II	0.76 (0.72‐0.80)	<0.001	0.82 (0.58‐1.17)	0.28
III	0.84 (0.77‐0.93)	<0.001	1.43 (1.02‐1.99)	0.037
IV	0.58 (0.52‐0.64)	<0.001	1.44 (1.04‐2.00)	0.027
Stage N				
0	Reference		Reference	
1	1.09 (1.03‐1.16)	0.004	1.67 (1.54‐1.82)	<0.001
2	1.49 (1.34‐1.66)	<0.001	2.53 (2.21‐2.90)	<0.001
3	1.15 (1.02‐1.30)	0.024	2.50 (2.14‐2.92)	<0.001
Stage M				
0	Reference		Reference	
1	0.28 (0.24‐0.32)	<0.001	0.47 (0.39‐0.57)	<0.001
Tumor size (cm)				
<2.0	Reference		Reference	
2.0‐5.0	0.76 (0.72‐0.81)	<0.001	1.04 (0.73‐1.48)	0.842
>5.0	0.73 (0.67‐0.78)	<0.001	1.23 (0.90‐1.69)	0.198
Chemotherapy				
No/unknown	Reference		Reference	
Yes	2.27 (2.13‐2.42)	<0.001	2.79 (2.58‐3.02)	<0.001
Surgery type				
No surgery	Reference		Reference	
Partial mastectomy	54.10 (42.37‐69.07)	<0.001	86.46 (66.72‐112.04)	<0.001
Total mastectomy	5.45 (4.24‐7.00)	<0.001	6.97 (5.36‐9.05)	<0.001
MRM	17.45 (13.62‐22.35)	<0.001	15.55 (12.04‐20.09)	<0.001

MRM, Modified radical mastectomy; OR, odds ratio.

### 3.3 Survival analysis of all population

Of the 22 802 patients finally recruited, 3446 patients were dead at the end of the last follow‐up. Moreover, 2749 patients were dead from breast cancer specifically. The Kaplan‐Meier plots displayed that patients in the radiation group had better survival than the no radiation group in both BCSS and OS (*P* < 0.001, respectively). The survival curves of BCSS and OS are exhibited in Figure 2.

**Figure 2:** Survival curves with the log‐rank tests of (A) breast cancer‐specific survival (*P* < 0.001) and (B) overall survival (*P* < 0.001)

The Cox proportional hazard model was applied to further probe the effect of multiple factors on BCSS and OS. In univariate analysis of BCSS, higher grade, more advanced TNM stage, larger tumor size, were proved to be risk factors for poor survival (HR > 1, *P* < 0.001). By contrast, age 40‐60, married status, white and other race, chemotherapy, radiation, and surgery were found to be protective factors for better survival (HR < 1, *P* < 0.05). Specifically, patients who received radiotherapy exhibited better BCSS (hazard ratio [HR] = 0.52, 95% CI = 0.48‐0.57, *P* < 0.001). All these variables mentioned above were subsequently enlisted in the multivariate Cox analysis. After adjusting for those confounding factors above, receipt of radiotherapy was still associated with improved BCSS (hazard ratio [HR] = 0.79, 95% CI = 0.72‐0.87, *P* < 0.001), compared with the no radiation group (Table 3). The detailed results of Cox regression analysis of BCSS are available in Table 3. Similarly, univariate analysis of OS also indicated that radiation was associated with a significant survival advantage over the no radiation group (HR = 0.50, 95% CI = 0.47‐0.54, *P* < 0.001). In multivariate Cox regression analysis, those patients treated with radiotherapy had superior OS (HR = 0.76, 95% CI = 0.70‐0.82, *P* < 0.001) compared to those not radiated (Table 4). The concrete results of OS analysis are shown in Table 4. Generally, these data indicate that radiotherapy after surgery has significant survival benefits for the whole TNBC patients.

**Table 3:** Cox proportional hazard regression model of breast cancer‐specific survival (n = 22 802)

Characteristics	Univariate Cox		Multivariate Cox	
	HR (95% CI)	*P* value	HR (95% CI)	*P* value
Age (y)				
<40	Reference		Reference	
40‐60	0.84 (0.74‐0.95)	0.007	0.98 (0.87‐1.12)	0.794
>60	1.06 (0.94‐1.20)	0.325	1.23 (1.08‐1.40)	0.01
Marital status				
Not married	Reference		Reference	
Married	0.62 (0.57‐0.66)	<0.001	0.82 (0.76‐0.88)	<0.001
Race				
Black	Reference		Reference	
White	0.74 (0.68‐0.81)	<0.001	0.98 (0.89‐1.07)	0.619
Others	0.63 (0.53‐0.74)	<0.001	0.76 (0.64‐0.90)	0.002
Grade				
I	Reference		Reference	
II	2.31 (1.51‐3.55)	<0.001	1.78 (1.16‐2.73)	0.009
III	2.98 (1.96‐4.53)	<0.001	2.24 (1.47‐3.42)	<0.001
IV	4.35 (2.58‐7.31)	<0.001	2.46 (1.46‐4.14)	0.001
Stage T				
I	Reference		Reference	
II	2.68 (2.40‐3.00)	<0.001	2.29 (1.70‐3.08)	<0.001
III	7.22 (6.36‐8.20)	<0.001	2.66 (2.00‐3.51)	<0.001
IV	16.72 (14.82‐18.86)	<0.001	3.76 (2.88‐4.91)	<0.001
Stage N				
0	Reference		Reference	
1	3.54 (3.23‐3.88)	<0.001	2.07 (1.87‐2.29)	<0.001
2	5.41 (4.80‐6.10)	<0.001	2.86 (2.50‐3.27)	<0.001
3	10.64 (9.52‐11.89)	<0.001	3.37 (2.95‐3.85)	<0.001
Stage M				
0	Reference		Reference	
1	15.95 (14.63‐17.39)	<0.001	4.19 (3.76‐4.67)	<0.001
Tumor size (cm)				
<2.0	Reference		Reference	
2.0‐5.0	2.52 (2.26‐2.80)	<0.001	0.87 (0.66‐1.15)	0.335
>5.0	8.37 (7.52‐9.32)	<0.001	1.27 (0.99‐1.64)	0.058
Chemotherapy				
No/unknown	Reference		Reference	
Yes	0.90 (0.83‐0.98)	0.013	0.57 (0.52‐0.63)	<0.001
Radiation				
No	Reference		Reference	
Yes	0.52 (0.48‐0.57)	<0.001	0.79 (0.72‐0.87)	<0.001
Surgery type				
No surgery	Reference		Reference	
Partial mastectomy	0.08 (0.07‐0.08)	<0.001	0.35 (0.30‐0.40)	<0.001
Total mastectomy	0.11 (0.10‐0.13)	<0.001	0.37 (0.33‐0.43)	<0.001
MRM	0.27 (0.24‐0.29)	<0.001	0.48 (0.43‐0.54)	<0.001

HR, hazard ratio; MRM, Modified radical mastectomy.

**Table 4:** Cox proportional hazard regression model of overall survival (n = 22 802)

Characteristics	Univariate Cox		Multivariate Cox	
	HR (95% CI)	*P*‐value	HR (95% CI)	*P*‐value
Age (y)				
<40	Reference		Reference	
40‐60	0.90 (0.79‐1.01)	0.069	1.04 (0.92‐1.17)	0.579
>60	1.39 (1.24‐1.57)	<0.001	1.50 (1.33‐1.69)	<0.001
Marital status				
Not married	Reference		Reference	
Married	0.57 (0.54‐0.61)	<0.001	0.77 (0.72‐0.83)	<0.001
Race				
Black	Reference		Reference	
White	0.77 (0.71‐0.83)	<0.001	0.97 (0.90‐1.05)	0.47
Others	0.63 (0.54‐0.73)	<0.001	0.75 (0.64‐0.88)	<0.001
Grade				
I	Reference		Reference	
II	2.15 (1.51‐3.08)	<0.001	1.78 (1.25‐2.55)	0.002
III	2.53 (1.79‐3.59)	<0.001	2.19 (1.54‐3.11)	<0.001
IV	3.59 (2.30‐5.62)	<0.001	2.37 (1.51‐3.72)	<0.001
Stage T				
I	Reference		Reference	
II	2.30 (2.09‐2.52)	<0.001	2.26 (1.73‐2.95)	<0.001
III	5.45 (4.88‐6.09)	<0.001	2.55 (1.98‐3.27)	<0.001
IV	12.51 (11.27‐13.88)	<0.001	3.58 (2.82‐4.55)	<0.001
Stage N				
0	Reference		Reference	
1	2.85 (2.63‐3.08)	<0.001	1.88 (1.72‐2.06)	<0.001
2	4.29 (3.86‐4.78)	<0.001	2.60 (2.31‐2.93)	<0.001
3	8.10 (7.32‐8.95)	<0.001	3.07 (2.72‐3.46)	<0.001
Stage M				
0	Reference		Reference	
1	12.70 (11.71‐13.78)	<0.001	3.67 (3.31‐4.06)	<0.001
Tumor size (cm)				
<2.0	Reference		Reference	
2.0‐5.0	2.20 (2.01‐2.41)	<0.001	0.83 (0.64‐1.07)	0.149
>5.0	6.45 (5.88‐7.07)	<0.001	1.18 (0.94‐1.48)	0.151
Chemotherapy				
No/unknown	Reference		Reference	
Yes	0.66 (0.61‐0.71)	<0.001	0.48 (0.44‐0.51)	<0.001
Radiation				
No	Reference		Reference	
Yes	0.50 (0.47‐0.54)	<0.001	0.76 (0.70‐0.82)	<0.001
Surgery type				
No surgery	Reference		Reference	
Partial mastectomy	0.09 (0.08‐0.10)	<0.001	0.37 (0.33‐0.42)	<0.001
Total mastectomy	0.14 (0.12‐0.15)	<0.001	0.40 (0.36‐0.46)	<0.001
MRM	0.28 (0.26‐0.31)	<0.001	0.50 (0.45‐0.55)	<0.001

HR, hazard ratio; MRM, Modified radical mastectomy.

### 3.4 Survival analysis stratified by T stage

To better understand the survival benefits of radiotherapy after surgery for the TNBC patients, we further analyzed the influence of radiotherapy on patients' survival stratified by T stage. The Kaplan‐Meier plots indicated that radiation exerted BCSS benefits for patients from both T1‐T2 population and T3‐T4 population (*P* < 0.001, respectively). Apparently, the survival benefits for T3‐T4 patients appeared more remarkable. The survival curves of BCSS analysis stratified by T stage are displayed in Figure 3.

**Figure 3:** Survival curves with the log‐rank tests of breast cancer‐specific survival for T1‐T2 population (A) and T3‐T4 population (B)

### 3.5 Survival analysis stratified by surgery type

Given surgery approaches may also affect radiation strategies. For solid elucidation of the survival benefits from radiotherapy after different surgery types, we stratified those patients by surgery type for further survival analysis. As is shown in Figure 4A, radiation exerted a significant survival advantage for patients after partial mastectomy. By contrast, radiation exerted significant survival disadvantage for patients after total mastectomy (Figure 4B). Furthermore, radiation had no significant survival benefit for patients after modified radical mastectomy (Figure 4C). Consequently, different surgery types may also affect the influence of radiotherapy on the survival of TNBC patients.

**Figure 4:** Survival curves with the log‐rank tests of breast cancer‐specific survival for partial mastectomy (A), total mastectomy (B), and modified radical mastectomy (C)

## 4 DISCUSSION

Currently, controversies regarding the use of radiotherapy for TNBC may affect decisions for the locoregional management of those patients.^9^ Based on a large population from the SEER database, this study retrospectively examined the clinicopathological characteristics and the efficacy of radiotherapy on survival outcomes of TNBC patients. Our data indicate that radiotherapy after surgery provided significant survival benefits of both BCSS and OS for the TNBC patients.

The value of adjuvant radiotherapy for TNBC has been appraised by several previous reports. A retrospective analysis of breast cancer patients from the Danish Breast Cancer Cooperative Group (DBCG) 82b and 82c trials revealed no survival benefit for postmastectomy radiation within TNBC patients.^10^ This study only enrolled 152 TNBC patients, limiting the power of the analysis. Comparatively, our investigation has recruited a much larger population of TNBC patients. So the power of analysis in our study seems more convincing. On the other hand, another recent study reported that adjuvant radiotherapy appeared to be independently associated with a survival gain in locally advanced as well as in very young TNBC.^11^ Consistent with this study, our results reflected that patients received radiotherapy after surgery exhibited better BCSS and OS in Kaplan‐Meier plots and Cox regression analysis. Moreover, we also analyzed the clinicopathological factors associated with receipt of radiotherapy. The multivariate logistic analysis revealed that married status, stage T3‐T4, stage N1‐N3, received chemotherapy, and surgery were independent factors associated with receipt of radiotherapy. These findings may help us to select the potential population who will benefit from post‐surgery radiation.

Nevertheless, radiotherapy did not appear to be constantly associated with an overall survival benefit in TNBC.^12^ In addition to radiotherapy after surgery, several confounding factors such as age at diagnosis, marital status, tumor TNM stage, chemotherapy may also account for the potentially important survival differences. In order to adjust the confounding variables of baseline demographic, clinicopathological, and treatment characteristics, we applied multivariate Cox regression analysis to highlight the influence of radiotherapy on the survival of TNBC patients. Our results reflected that women received radiotherapy after surgery exhibited better BCSS and OS than those without radiation in multivariate Cox regression analysis after adjusting for confounding variables. So our findings are in accordance with Chen's study, which claimed that TNBC patients treated with postmastectomy radiotherapy significantly improved survival in the entire cohort.^13^ Our findings uphold the recommendation of radiotherapy for TNBC patients after surgery.

Although we have found the significant survival benefits from radiotherapy after surgery based on all population analysis, the majority of patients included were pT1‐2N0‐1. For solid elucidation, we stratified those patients by T stage for further survival analysis. The subgroup analysis indicated that radiation exerted BCSS benefits for patients from both T1‐T2 population and T3‐T4 population. Comparatively, the previous study reported that T1‐2N0 TNBC treated with modified radical mastectomy without radiotherapy had a significantly increased risk of locoregional recurrence and poorer survival.^7^ So our results have highlighted the vital role of radiotherapy for the TNBC patients after surgery. In addition, different surgery types may also affect the influence of radiotherapy on the survival of TNBC patients, so we have performed further stratified analysis by surgery types. Intriguingly, the overall results indicated that radiotherapy only exerted significant survival advantage for patients after partial mastectomy rather than those after total mastectomy or MRM. These findings are consistent with previous reports, which revealed that breast conservation therapy with radiotherapy produced significant survival advantage over MRM or mastectomy only.^7^, ^11^ As a result, the evidence of radiation following breast conservation therapy has become more adequate from our study.

Inevitably, there are several limitations to our study. First, this is a retrospective study from SEER database rather than a prospective cohort study, so the inherent selection biases could limit the external validity of this study. Second, information about cancer recurrence and subsequent sites of disease involvement is not available from SEER database, so we are unable to evaluate the influence of radiotherapy on locoregional recurrence‐free survival of the patients. Third, SEER database does not provide detailed information about radiotherapy (site, extent, and technique‐stereotactic radiosurgery or whole‐brain radiotherapy). These variables may also affect the survival of TNBC patients. These limitations may have contributed to study bias and undermine the power of analysis.

## 5 CONCLUSION

In conclusion, our study indicates that radiotherapy after surgery has significant survival benefits for the patients with TNBC. The survival advantage of adjuvant radiotherapy for TNBC patients has been confirmed in this study. Our results may optimize the current individualized treatment decisions for the TNBC patients. Further prospective clinical trials are still needed to validate our findings.

## CONFLICT OF INTEREST

The authors declare no conflicts of interest in this work.
